# The Effect of Mesenchymal Stromal Cells on the Mortality of Patients with Sepsis and Septic Shock: A Promising Therapy

**DOI:** 10.1155/2022/9222379

**Published:** 2022-06-24

**Authors:** Emine Alp, Zeynep Burcin Gonen, Kursat Gundogan, Aliye Esmaoglu, Leylagul Kaynar, Aysun Cetin, Musa Karakukcu, Mustafa Cetin, Gamze Kalin, Mehmet Doganay

**Affiliations:** ^1^Department of Infectious Diseases and Clinical Microbiology, Medical Faculty, Ankara Yıldırım Beyazıt University, Ankara, Turkey; ^2^Oral and Maxillofacial Surgery, Genome and Stem Cell Center (GENKOK), Erciyes University, Kayseri, Turkey; ^3^Medical Intensive Care Unit, Department of Internal Medicine, Faculty of Medicine, Erciyes University, Kayseri, Turkey; ^4^Department of Anesthesiology and Reanimation, Faculty of Medicine, Erciyes University, Kayseri, Turkey; ^5^Bone Marrow Transplant and Stem Cell Unit, Division of Hematology, Department of Internal Medicine, Faculty of Medicine, Erciyes University, Kayseri, Turkey; ^6^Department of Biochemistry, Faculty of Medicine, Erciyes University, Kayseri, Turkey; ^7^Division of Pediatric Hematology and Oncology, Department of Pediatrics, Faculty of Medicine, Erciyes University, Kayseri, Turkey; ^8^Department of Infectious Diseases and Clinical Microbiology, Faculty of Medicine, Erciyes University, Kayseri, Turkey; ^9^Department of Infectious Diseases, Faculty of Medicine, Lokman Hekim University, Ankara, Turkey

## Abstract

**Purpose:**

Sepsis and septic shock are the major causes of death in intensive care units. This study aimed to evaluate the clinical safety and efficacy of mesenchymal stem cells (MSCs) in sepsis and septic shock patients.

**Methods:**

Ten patients were enrolled in the study. Adipose-derived MSC infusions were given (1 × 10^6^/kg, on the 1^st^, 3^rd^, 5^th^, 7^th^, and 9^th^ days of therapy) together with standard therapy. Before the MSC applications, blood samples were collected for cytokine assessment (TNF-*α*, IFN-*γ*, IL-2, IL-4, IL-6, IL-10). The clinical and laboratory improvements were recorded and compared with control groups selected retrospectively. The clinical trial was registered on 16.03.2022 with the registration number NCT05283317.

**Results:**

In the study group, the ages of patients ranged from 22 to 68 years, and APACHE II scores ranged from 14 to 42. In the control group, ages ranged from 22 to 80 years and their APACHE II scores were between 14–35. The survival rate in the study group was 100% on the 14^th^ day whereas it was 70% on the 28^th^ day. A significant decrease in the SOFA score (adjusted), clinical, and laboratory improvements were observed during the MSC administration. However, no significant cytokine level changes were observed. In the control group, the survival rate of 20 patients was 70% on the 14^th^ day, whereas 60% was on the 28^th^ day. While deaths were observed in the control group in the first week of treatment, deaths in the MSCs group were observed between the 15^th^ and 28^th^ days.

**Conclusion:**

MSCs treatment may have a positive impact on the survival rates of sepsis during the early phase. However, further randomized controlled studies with a large group of patients are needed. *Trial Registration*. This trial is registered with ClinicalTrials.gov Identifier: NCT05283317.

## 1. Introduction

Sepsis is defined as an immune response that paves the way for microcirculatory and endothelial cell dysfunction, leading to multiple organ dysfunction, which is the most common cause of mortality and critical illness in hospitalized patients. Sepsis and septic shock are still serious public health problems with increasing incidence by year and year with high mortality. Moreover, it has an important socioeconomic impact on the health system of countries [1].

It is reported that the incidence of sepsis has been increasing over the years in developed countries. Approximately 750000 people in the US are diagnosed with sepsis, and the number of estimated deaths from sepsis reaches a quarter of a million per year [2, 3]. Although the actual incidence of sepsis in developing countries is not known completely, it is thought that the incidence of sepsis accounts for 2% to 11% of hospitalizations and intensive care unit admissions [4]. The number of reported incidences of sepsis is rising due to changes in patients' demography, advanced age, more comorbidities, impaired immunity, and recognition of sepsis [3]. Furthermore, survivors of sepsis have a higher mortality rate in the five years after the sepsis experience; they also suffer from cognitive, physical, and psychological impairments [3].

There are many research studies for new pharmacological agent studies to decrease the mortality rate associated with sepsis. At this point, stem cell therapy, which is shown as the most important development in recent years, may result in positive effects on some diseases such as autoimmune diseases, transplantation, surgery, and sepsis. Therefore, stem cells, currently used for pathologies such as autoimmune disease, transplantation, and surgery, could be helpful in the management of patients with sepsis. The mortality rate is reported to be between 20% and 80%, and it is higher at advanced age and with concomitant diseases [5–8]. It has been reported that the mortality rates depend on the severity of infection and sepsis stage; the mortality rate is 0–36% in sepsis, 18–52% in severe sepsis, and 46–82% in septic shock [9, 10].

Currently, the main therapy of sepsis consists of antibiotics therapy, other supportive therapies, and source control of infection, but no sufficient agents are reducing the systemic inflammation and organ dysfunctions in sepsis [11]. Early detection with timely administration of antibiotics and fluids has encouraging results on mortality. However, these effects are not satisfying for clinicians, and new therapies are still needed. At this point, stem cell therapy, which is shown as the most important development in recent years, may result in positive effects on some diseases such as autoimmune diseases, transplantation, surgery, and sepsis [12].

Mesenchymal stem cells (MSCs) are multipotent cells with the capacity to differentiate into cells from all three lineages, and they constitute a therapeutic potential for sepsis. It can be indicated that MSCs are popular candidates for sepsis therapy because of their immune-privileged nature and the potential to alter sepsis pathophysiology. First of all, MSCs are relatively immune-privileged due to the low human leukocyte antigen (HLA) class I and II expression levels. Therefore, MSCs can be used as an allogeneic therapy without any immunosuppression protocol for the patient. Secondly, they weaken various aspects of the immune response to sepsis; MSCs form a more complex immune action profile. MSCs can reprogram the immune system to reduce host tissue damage while maintaining the immune response against microorganisms. Thirdly, MSCs can enhance tissue repair and restoration after sepsis; they can restore endothelial barrier function, partially mediated by paracrine factors that affect the microenvironment of tissue damage. Fourthly, sepsis and septic shock cause dysfunction and failure of multiple organs. In this respect, MSCs can reduce injury and/or reduce and restore function in various organs because of their antimicrobial and anti-inflammatory features [11]. Fifthly, MSCs can directly increase host bactericidal capacity by increasing macrophage bacterial phagocytosis and increasing the secretion of antimicrobial peptides. Sixthly, MSCs are being well studied with an increased safety record in patients in clinical trials [3, 11].

They have a capacity for cytokine secretion to differentiate along various lineages, immune modulation, and direct cell-cell interaction with damaged tissue. In sepsis, endothelial damage is the main pathogenic mechanism that leads to organ damage and mortality. Many experimental animal studies of sepsis have been carried out and the results are showing the beneficial effect of MSCs on the survival rate. In these studies, the contribution of MSCs to survival may be related to the mechanism of anti-inflammatory and immunomodulatory effects [13, 14]. However, published evidence from clinical trials approving the efficiency and safety of MSCs in humans with septic shock is very limited [15]. There are ongoing clinical trials that are registered in trial databases such as SEPCELL, CHOCMSC, CISS2, and RUMCESS trials [16–19].

In this respect, this study aims to assess the safety of five doses of application of adipose-derived MSCs on the mortality of patients with sepsis and septic shock.

## 2. Patients and Methods

### 2.1. Study Design and Setting

The study was carried out at the Internal Medicine Intensive Care Unit (IMICU) and the Anesthesiology and Reanimation Intensive Care Unit (ARICU) at Erciyes University Hospital which is a referral hospital in Central Anatolia. The study was approved by the Erciyes University Ethics Board (2016/114; Date: 19.02.2016) and the Ministry of Health of Turkey. Informed consent from surrogate decision-makers was obtained for study participation after confirmation of eligibility criteria. The clinical trial was registered on 16.03.2022 with the registration number NCT05283317 [20].

### 2.2. Patients

The study was planned prospectively. For two years, 10 patients with sepsis and septic shock were included in the study from IMICU and ARICU. Sepsis and septic shock were diagnosed according to the sepsis guidelines [1]. Inclusion criteria for this study were as follows: patients who were between 18 and 80 years of age and were hospitalized at IMICU and ARICU with the diagnosis of sepsis and septic shock. Exclusion criteria were categorized as follows: patients who were younger than 18 years and older than 80 years and were pregnant women or breastfeeding, patients who had a terminal stage of cancer, advanced pulmonary disease receiving oxygen at home, advanced pulmonary hypertension (WHO Class III or IV), advanced heart failure (American Heart Association Class III or IV), severe liver disease (Child C), and history of anaphylaxis. Standard therapy of sepsis as suggested in the guidelines [1, 2] was given to all patients, and additionally, MSC treatment was applied to the patients in the study group. Control patients diagnosed with sepsis and septic shock and having similar characteristics for the consideration of the severity of the disease based on APACHE II score and comorbid diseases to the study group were selected from IMICU and ARICU records retrospectively.

Patients' demographic characteristics, underlying diseases, and clinical and laboratory outcomes were recorded.

### 2.3. Source and Applications of MSCs

MSCs were prepared in the Good Manufacturing Practices (GMP) Laboratory of the Genome and Stem Cell Center at Erciyes University. Cell production and quality control assessment procedures were carried out according to GMP protocols authorized by the Ministry of Health of Turkey. Allogenic adipose-derived MSCs (ADMSCs), which were obtained from a healthy donor, were applied to all patients in the study group. Five doses of ADMSCs were applied to the patients on the 1^st^ and 3^rd^ days (postthawed of frozen MSCs, cryo-bag), 5^th^-7^th,^ and 9^th^ days (replated ADMSCs vials) of therapy. Each dose of ADMSCs was prepared as 1 × 10^6^ ADMSCs/kg. The vials containing ADMSCs were mixed with gentle motion before usage; thus, it ensured product homogenization. ADMSCs were infused intravenously via a central venous line in a physiological saline solution by using a blood transfusion set. The patients were monitored during all these procedures.

### 2.4. Preparation of ADMSCs

Sufficient cryopreserved ADMSC vials were thawed to provide the required dose for administration. The frozen ADMSCs were thawed and cultured in Dulbecco's modified Eagle's medium (DMEM) containing 10% human serum, 1% penicillin-streptomycin solution, and 1% stable glutamine (Biological Industries, Kibbutz Beit Haemek, Israel) at 37°C and 5% CO_2_ incubator as described before [16]. Briefly, ADMSCs were recovered and resuspended in physiological saline solution and transferred to the patient with the temperature-controlled bag. The morphology of cell appearance and viability were assessed besides the identification of phenotypic characteristics of the cells and microbiological tests. Immunophenotyping characterization of ADMSC was performed by using flow cytometry analyses (Beckman Coulter, USA) with antibodies against CD45, CD73, CD90, CD105, CD11b, CD19, CD34, and CD44 (BD Stem Flow hMSC kit).

### 2.5. Cytokine Analysis

10 ml of peripheral venous blood samples was collected before each MSC infusion on the 1^st^, 3^rd^, 5^th^, 7^th^, and 9^th^ days of therapy. The serum samples were centrifuged at 5000 rpm for 5 minutes and stored at −80°C until laboratory analysis. The cytokine level was analyzed with the ELISA method by using Human BioSource for IFN-*γ*, IL-2, IL-4, and IL-10 kits in the Robonik Read Touch model (Robonik India Pvt. Ltd) device.

### 2.6. Clinical and Laboratory Follow-Up

Clinical findings and laboratory results were recorded during the administration of MSCs infusions on the 1^st^, 3^rd^, 5^th^, 7^th^, and 9^th^ days. Patients' demographic characteristics, underlying diseases, and clinical and laboratory outcomes were recorded. The patients were monitored for unexpected adverse events. In the clinical follow-up of the patient's APACHE II, SOFA (sequential organ failure assessment score) score, clinical progression, and outcome of patients were recorded. In the laboratory, the following inflammatory markers were also recorded: C reactive protein (CRP), procalcitonin (PCT), white blood cell (WBC), bleeding parameters (platelets, INR, fibrinogen), lactate, liver enzymes (AST, ALT), and renal function (creatinine). Laboratory test results were analyzed according to MSCs administration days. The differences in the laboratory tests were compared between the survivor and nonsurvivor patients according to MSCs therapy days.

The outcomes of the patients were compared with the previous observational study conducted in the same Intensive Care Units (ICUs) as the control. The day of death and 0–6^th^, 7–14^th^, and 15–28^th^ days were determined as survival status and endpoint. In the case of death, the date and cause of death were also recorded.

### 2.7. Statistical Analysis

In the study, the results were compared to controls. Statistical analysis was performed using the Turcosa software. The relationships between categorical variables were analyzed by chi-square analysis. When parametric assumptions were provided in the comparison of numerical variables in the two groups, the Student *T*-test was used, and the Mann–Whitney *U*-test was used in the case that the parametric assumptions were not provided. For the analysis of repeated measurements, the paired sample *T*-test was used for binary comparisons, and the repeated-measures ANOVA test was used for comparisons of more than two repeated measurements. The survival probability of the patients during the follow-up period was determined by the Kaplan–Meier survival analysis. The effects of age and APACHE II on covariant analysis were adjusted. *p* < 0.05 was accepted as statistically significant.

## 3. Results

### 3.1. Morphology and Phenotype of ADMSCs

ADMSCs were adherent to the plate during cell culture. The cells had a spindle-shaped morphology. No evidence of bacterial or fungal contamination was observed in the cells which were tested before release. The mean cell viability was found to be 92.2% ± 2.5 before cell infusion. The ADMSCs were found positive for CD44 (%95.7 ± 2.1), CD73 (%96.6 ± 2.5), CD90 (%97.5 ± 2.1), and CD105 (96.4% ± 2.8) and negative for CD11b, CD34, CD45, and HLA-DR (0.3% ± 0.2) (Figure 1).

### 3.2. Patients

The study group consisted of 6 males and 4 females, aged between 22 and 68 years, and 7/10 (70%) patients had at least one underlying disease with APACHE II scores ranging from 14 to 42. The sources of sepsis were urinary tract infection in 3 patients, pneumonia in 2, abdominal infection in 2, meningoencephalitis in 1, pancreatitis in 1, and bacteremia in 1.

The control group consisted of 20 patients with sepsis and septic shock who were followed in the same ICU and whose clinical features were similar to the study group. It consisted of 15 males and 5 females aged between 22 and 80 years, and 17/20 (85%) patients had at least one underlying disease with APACHE II scores ranging from 14 to 35. The majority of the sources of sepsis were the respiratory system in the control group. Patients in the control group were older; however, respiratory failure was more common and creatinine levels were higher in the study group (Table 1).

In the study group, the survival rate was 100% on the 7^th^ and 14^th^ days, while the rate decreased to 70% on the 28^th^ day. A significant decrease in the SOFA score in the MSCs treatment group, which was adjusted by age and APACHE II, was found by the treatment days (*p*=0.027).

No MSC infusion-associated or unexpected serious adverse events were observed during the study period and follow-up 28^th^ day.

In the control group, the survival rate of 20 patients was 60% on the 28^th^ day. The difference between the groups was not statistically significant. However, deaths were observed in the control group before the 7^th^ day of treatment, and no deaths were observed in the MSC treatment group for the first two weeks and during the period of MSC administration. Deaths in the study group were observed between the 15^th^ and 28^th^ days. The causes of death of these three patients were that one of them had prolonged mechanical ventilation due to nosocomial infection, the other one had metastatic malignancy, and the third patient developed intracranial infarction. On the other hand, the hospital stay of the patients in the study group was longer than that in the control group, but the difference was not significant (*p*=0.091).

### 3.3. Laboratory Results of the Patients

In the study group, the initial CRP and PCT values were significantly higher than in the control group. However, there was no difference between the two groups on the fifth and 14^th^ days of follow-up (Table 2).

In the study group, CRP and WBC were significantly lowered at the end of the treatment period according to the initial values (*p* − CRp=0.028; *p* − WBc=0.045). Although there were improvements in the laboratory findings (PCT, lactate, and platelets) during the MSC applications, the improvements were not statistically significant (*p* > 0.05). Cytokine levels, which were compared to the basal measurement on the 1^st^, 3^rd^, 5^th^, and 7^th^ days, were also not significant (Table 3).

There was no statistically significant difference when the laboratory results of the survivors and nonsurvivors were compared on the 1^st^, 5^th^, and 14^th^ days in the study group. However, CRP and PCT levels were higher in the patients who died on the indicated days. Platelet values were lower in patients who died compared with the survivors on the 14^th^ day. No significant difference was found between the cytokine values of the survivor and nonsurvivor patients (Table 4).

## 4. Discussion

MSCs have assumed a therapeutic potential effect on sepsis and septic shock, which was shown in previous limited clinical studies [21, 22]. Many experimental animal studies of sepsis have been carried out and have shown the beneficial effect of MSC treatment on survival [13, 23–25]. In current clinical studies, the average mortality rate of sepsis has been reported as 50% [26]. He et al. (2018) showed that this rate was 20% in patients with sepsis undergoing single-dose MSC treatment. In the present study, no deaths were observed in the study group for the first two weeks and the period of MSC administration. It is known that MSCs have a therapeutic effect on sepsis with their anti-inflammatory and immunomodulatory effects [27], and this effect may have a positive impact on survival.

The determination of the optimal dose of MSCs to treat patients with sepsis and septic shock is debatable. This determination process is difficult due to three reasons: (1) limitations in existing dosing data in humans; (2) variability in human biologic measurements in septic shock; and (3) a potential lack of conformity of cell therapy to the dose-response relationship that is common with pharmaceutical drugs [15]. He et al. (2018) conducted a clinical study in China by using umbilical cord-derived MSCs of 3 different doses (1 million/kg, 2 million/kg, and 3 million/kg) on the effect of five patients, which was investigated [22]. This study showed that the single dose of allogeneic 3 million/kg cells was safe and well tolerated by the patients. In the present study, allogeneic ADMSCs induced by five doses of 1 million/kg were well tolerated and no side effects were observed in ten cases.

APACHE II shows a score of the severity of the infection and the outcome of sepsis. It is reported that in sepsis patients with high APACHE II scores, the expected mortality is over 50%, and they are considered high-risk patients for mortality [28]. Therefore, other treatments based on the pathogenesis of sepsis are needed in addition to standard sepsis treatment to increase survival rates in sepsis and septic shock [29, 30].

When the cytokine levels of survivors and nonsurvivors for the first 14 days were compared in Table 4, it is remarkable that the levels of proinflammatory IFN-*γ* and TNF-*α* decreased in surviving patients with MSC application. The same cytokines indicated an apparent quantitative increase in nonsurvivors. Considering these results, the rise in IFN-*γ* and TNF-*α* levels in nonsurvivors could be considered poor prognostic markers for increased mortality. For an effective interpretation of changes in other cytokine levels, including especially the evaluation of IL-1 and IL-6, further studies with a higher number of cases together with control groups need to be carried out.

The mortality rate for the 7^th^ and 14^th^ days of the 10 patients who were administered MSCs was 0%, while the mortality rate for the 28^th^ day was 30%. In the control group, the mortality rate was 40%, and the majority of the deaths were observed before the 5^th^ and 7^th^ days of treatment.

Of the cytokines measured in the present study IL-2, IFN-*γ*, and TNF-*α* have proinflammatory and IL-4 and IL-10 have anti-inflammatory properties. Although not significant, a quantitative decrease was evident on the 3^rd^, 5^th^, and 7^th^ days of MSC application for TNF-*α*, and the 1^st^, 3^rd^, 5^th^, and 7^th^ days for IL-10 levels in patients (Table 3). Likewise, He et al. (2018) reported that biomarkers (IL-6, TNF-*α* and CRP) decreased on the 8^th^ day after MSC treatment. It is known that bacterial lipopolysaccharides bring about TNF-*α* release in septic shock [22]. On the other hand, TNF-*α* stimulates the release of IL-1, IL-2, and IL-8 [31]. In this study, a statistically significant decrease in CRP was detected between the beginning and the 14^th^ day of the patients from the study group. Nevertheless, no improvement was observed in the control group.

The multipotency of MSCs has importance in tissue engineering and therapeutic use in sepsis. When tissue hypoxia is present like in sepsis and septic shock, the cytoprotective effect of MSC increases. In addition to them, the expression of antiapoptotic proteins (Bcl-2) increases, while the expression of proapoptotic proteins (caspase) reduces. Thus, endothelial apoptosis is reduced and endothelial integrity is achieved [14, 23, 24, 26, 32–34]. Consequently, MSCs could be a promising adjunctive therapy in sepsis with the ability to repair tissue in injury. MSCs have been preferred in stem cell treatment due to their differentiation potential into many different cell types, regulation of immune response, proangiogenic and damage repairing features, low immunogenicity, and ease of production. Also, MSCs have an immunomodulatory role that modulates an immune response. The anti-inflammatory effect of MSCs has also been demonstrated. MSCs cause anti-inflammatory (growth factor-*β*, IL-10, IL-13) cytokine secretion and decrease the release of proinflammatory cytokines (TNF-*α*, IL-1, and IL-6). It is thought that the most important reason for the ineffectiveness of the previously anti-inflammatory cytokines in sepsis is that they affect a single stage of inflammation. It is expected that MSCs affect many stages of inflammation and show the cytoprotective effect; it leads to an increase in clinical success. However, in this study, the cytokines evaluated between survivors and nonsurvivors did not show statistically significant differences at the beginning. Moreover, the necessity of comparing the control group with cytokine values compatible with the patients is one of the limitations of our study. On the other hand, in the MSCs treatment group, a decrease in the SOFA score of the analyses, which were adjusted by age and APACHE II, was statistically significant compared with the control group (*p*=0.027).

The clinical use of MSCs has encountered many challenges including regulation and cell testing that need to be overcome worldwide. For the clinical development of MSCs as a potential treatment for septic shock, clinical cell processing and manufacturing problems must be solved. These problems involve the selection of an appropriate MSC dose, the determination of the optimal clinical outcomes, and the use of a fresh versus cryopreserved MSC product [15]. Therefore, the adaptation of cell therapy to clinical therapy has remained very limited. MSCs were safely studied in clinical trials involving approximately 1,000 patients with acute respiratory distress syndrome, but the safety of MSCs in septic shock was evaluated in only two studies with 27 patients and 9 patients with no safety issues [15]. The lack of an existing study on the safety and tolerability of MSCs for septic shock is also emphasized as one of the challenges in this issue, and future trials should be continued to evaluate the safety of MSCs in sepsis and septic shock [15].

The study has several limitations, and it was not a randomized controlled study. There were a limited number of patients included in the study compared with a retrospective control group, due to the project budget. There were differences in their characteristics (age, infection source, CRP, PCT, etc.), the lack of cytokine information in the control group, and the fact that patients receiving surviving MSC therapy required a longer ICU stay.

In conclusion, mesenchymal stem cell treatment is a promising therapy in sepsis and septic shock. The findings of this study suggest that MSC therapy is found to be a safe therapy in the early phase of sepsis and septic shock. These data are considered useful for further clinical studies on the effect and continuity of MSCs in the treatment of sepsis and septic shock. In the author's opinion, further collaborative, prospective, and randomized controlled clinical studies may be useful for highlighting the effect of MSCs on patients with sepsis and septic shock.

## Figures and Tables

**Figure 1:** Histogram of the ADMSCs (a) and the mean expression levels of the markers (b).

**Table 1:** The clinical characteristics of the mesenchymal stem cell (MSC) transplantation and comparison groups.

	MSC transplantation group (*n* = 10) *n* (%)	Control group (*n* = 20) *n* (%)	*P*
Baseline characteristics			
Age, median (min–max)	51 (22–68)	69 (22–80)	0.015
Male gender	6 (60.0)	15 (75.0)	0.675
Comorbid disease	7/10 (70%)	17/20 (85%)	0.633
APACHE II score, median (min–max)	27 (14–42)	28 (14–35)	0.779
SOFA score, median (min–max)	9 (2–18)	11 (4–18)	0.307

Qualifying organ failure, *n* (%)			
Respiratory failure	4 (40.0)	1 (5.0)	0.031
Renal failure	3 (30.0)	4 (20.0)	0.657
Coagulation failure	1 (10.0)	2 (10.0)	0.999
Organ hypoperfusion	9 (90.0)	11 (55.0)	0.101

Baseline organ failure (hypoperfusion)			
Renal, creatinine (mg/dL) median (min–max)	4.40 (0.21–7.80)	1.16 (0.26–8.07)	0.024
Hematologic, platelets (10^3^/*µ*L) median (min–max)	156000 (26000–479000)	200500 (18000–575000)	0.373
Liver enzyme (*μ*/L) median (min–max)			
Alanine aminotransferase (ALT) median	34 (3–861)	19 (5–1437)	0.713
Aspartate aminotransferase (AST) median	49 (19–158)	26 (10–2205)	0.231
Lactate (mmol/L) median (min–max)	1.42 (0.82–3.17)	1.69 (0.80–9.96)	0.350

Infectious source *n* (%)			
Lung	2 (20.0)	12 (60.0)	
Urinary	3 (30.0)	3 (15.0)	
Intraabdominal	3 (30.0)	5 (25.0)	0.063
Meningoencephalitis	1 (10.0)	0 (0.0)	
Bacteraemia	1 (10.0)	0 (0.0)	
ICU length of stay (survivors)			
Median (min–max)	26 (10–91)	10 (3–32)	0.001
Hospital length of stay (survivors)			
Median (min–max)	28 (16–91)	16 (5–40)	0.091

Clinical outcomes			
Mortality, *n* (%; 95% CI)			
14 day	0 (0.0)	6 (30.0)	0.141
28 day	3 (30.0)	8 (40.0)	0.702

**Table 2:** Comparison of changes in laboratory tests of ADMSCs treatment and control groups by days.

Laboratory tests	MSC transplantation group (*n* = 10)	Control group (*n* = 20)	*p*
*0 days*			
CRP (mg/mL)	207 (32–334)	100 (16–313)	0.031
PCT (mg/mL)	3.64 (0.65–100.0)	1.17 (0.07–24.0)	0.009
Laktat (mmol/L)	1.42 (0.82–3.17)	1.69 (0.80–9.96)	0.350
WBC (10^3^/*μ*l)	17100 (3070–41800)	12230 (680–24700)	0.074
AST (*μ*/L)	49 (19–158)	26 (10–2205)	0.231
ALT (*μ*/L)	34 (3–861)	19 (5–1437)	0.713
Platelet (10^3^/*μ*l)	156000 (26000–479000)	200500 (18000–575000)	0.373
*5 days*			
CRP (mg/mL)	82 (20–275)	64 (11–185)	0.562
PCT (mg/mL)	2.24 (0.48–100.0)	0.50 (0.40–1.78)	0.777
Laktat (mmol/L)	1.31 (0.63–2.84)	1.23 (0.54–2.54)	0.974
WBC (10^3^/*μ*l)	11190 (1990–40310)	9200 (3620–24400)	0.232
AST (*μ*L)	33 (10–88)	25 (10–56)	0.367
ALT (*μ*L)	25 (2–134)	14 (4–185)	0.643
Platelet (10^3^/*μ*l)	214000 (35000–925000)	159000 (19810–430000)	0.285
*14 days*			
CRP (mg/mL)	62 (22–295)	105 (84–36)	0.287
PCT (mg/mL)	1.21 (0.27–7.56)	1.14 (0.98–1.30)	0.909
Laktat (mmol/L)	1.44 (0.80–2.43)	0.93 (0.63–2.38)	0.181
WBC (10^3^/*μ*l)	9530 (1750–52230)	8150 (3490–13500)	0.274
AST (*μ*L)	31 (7–124)	36 (19–55)	0.768
ALT (*μ*L)	24 (4–169)	14 (13–21)	0.440
Platelet (10^3^/*μ*l)	190000 (40000–791000)	214000 (21000–385000)	0.813

ADMSCs: allogenic adipose-derived MSCs.

**Table 3:** Cytokine levels and laboratory results of the patients in the ADMSC group.

	Treatment days					*p*
	0	1	3	5	7	
*Cytokines*						
IL-2	42.1 (28.5–304.9)	76.0 (25.2–279.3)	71.8 (40.0–273.6)	59.0 (15.4–243.4)	59.3 (45.0–258.0)	0.516
IL-4	418.4 (4.3–2597.5)	298.8 (0.9–2639.8)	210.0 (54.2–2390.8)	280.8 (24.6–2602.5)	417.5 (25.4–2716.7)	0.404
IL-10	18.5 (0.4–81.7)	19.2 (9.6–84.3)	15.9 (0.9–79.9)	13.8 (8.2–83.0)	13.4 (7.5–89.9)	0.647
TNF-*α*	105.5 (35.2–557.7)	136.5 (68.7–564.8)	140.6 (59.1–549.5)	123.7 (59.1–612.7)	99.0 (8.7–545.4)	0.416
IF-*Ɣ*	150.1 (82.2–814.6)	166.0 (101.9–956.7)	169.9 (109.5–953.7)	172.2 (73.7–1029.4)	181.4 (85.5–992.5)	0.275
*Laboratory results*						
CRP (mg/mL)	207 (32–334)	129 (99–279)	96 (46–217)	82 (20–275)	75 (17–208)	0.028
PCT (mg/mL)	3.6 (0.7–100.0)	3.1 (1.2–50.0)	2.8 (1.3–10.0)	2.2 (0.5–100.0)	1.6 (0.5–56.0)	0.641
WBC (*µ*/L)	17100 (3070–41800)	14840 (2750–39470)	12715 (2820–46570)	11190 (1990–40310)	11440 (2210–36940)	0.045
Lactate (mmol/L)	1.43 (0.82–3.17)	1.40 (1.09–2.20)	1.33 (0.99–2.29)	1.30 (0.63–2.84)	1.30 (0.80–4.84)	0.170
SOFA score (adjusted)	3.02 ± 0.84	2.7 ± 0.83	2.48 ± 0.75	1.99 ± 1.08	2.2 ± 0.78	0.027^*∗∗*^ adjusted

**Table 4:** Comparison of the cytokine levels and laboratory results between survivor and nonsurvivor patients in ADMSCs treatment group.

	Survivors				Nonsurvivors			
	Days				Days			
	<7 (0 day)	7–14 (7 day)	14–28 (14. day)	*p*	<7 (0 day)	7–14 (7 day)	14–28 (14 day)	*p*
*Cytokines*								
IL-2	49.4 (28.5–304.9)	116.7 (45.3–258.0)	ND	0.497	34.8 (28.6–83.8)	50.1 (45.0–50.7)	ND	0.980
IL-4	405.8 (4.3–2597.5)	305.0 (25.4–2716.7)	ND	0.530	431.0 (395.8–483.3)	530 (210.0–677.5)	ND	0.802
IL-10	22.3 (0.4–81.7)	14.0 (9.3–89.9)	ND	0.891	14.7 (11.4–24.5)	9.4 (7.5–30.1)	ND	0.777
TNF-*α*	137.5 (35.2–557.7)	100 (8.7–545.4)	ND	0.985	66.6 (47.1–146.2)	87.5 (47.3–184.8)	ND	0.215
IF-*ɣ*	179.8 (88.2–814.6)	152.8 (85.5–992.5)	ND	0.394	105.8 (82.2–223.1)	210.1 (96.7–241.3)	ND	0.260
*Laboratory results*								
CRP (mg/ml)	206 (32–290)	53 (17–208)	49 (22–295)	0.113	313 (153–334)	174 (150–198)	199 (70–228)	0.665
PCT (mg/ml)	3.5 (0.7–100.0)	1.2 (0.5–56.0)	0.6 (0.3–7.6)	0.510	6.3 (1.9-100.0)	2.8 (2.7–2.9)	2.5 (1.3–4.0)	0.385
WBC (*µ*/L)	18700 (10950–41800)	11440 (6910–36940)	7900 (7500–52230)	0.200	13700 (3070–21780)	7550 (2210–12890)	11160 (1750–12050)	0.386
Lactate (mmol/L)	1.5 (0.8–3.2)	1.3 (0.8–2.7)	1.8 (0.8–2.4)	0.583	1.4 (1.0–207)	2.9 (0.9–4.8)	1.4 (1.1–1.4)	0.588
Platelet (10^3^ /*μ*l)	150000 (26000–479000)	247000 (35000–925000)	324000 (40000–791000)	0.319	166000 (121000–266000)	172000 (118000–194000)	88000 (80000–124000)	0.381

ND: not done; ADMSCs: allogenic adipose-derived MSCs.

## Data Availability

The datasets generated during the current study are not publicly available as they contain health-related data, but limited datasets (without any identifiable person-related data) are available from the corresponding author upon reasonable request.

## References

[1] Singer M., Deutschman C. S., Seymour C. W. (2016). The third international consensus definitions for sepsis and septic shock (Sepsis-3). *JAMA*.

[2] Martin-Loeches I., Levy M., Artigas A. (2015). Management of severe sepsis: advances, challenges, and current status. *Drug Design, Development and Therapy*.

[3] Keane C., Jerkic M., Laffey J. G. (2017). Stem cell-based therapies for sepsis. *Anesthesiology*.

[4] Tupchong K., Koyfman A., Foran M. (2015). Sepsis, severe sepsis, and septic shock: a review of the literature. *African Journal of Emergency Medicine*.

[5] Munford R. S. (2006). Severe sepsis and septic shock: the role of gram-negative bacteremia. *Annual Review of Pathology: Mechanisms of Disease*.

[6] Esel D., Doganay M., Alp E., Sumerkan B. (2003). Prospective evaluation of blood cultures in a Turkish university hospital: epidemiology, microbiology and patient outcome. *Clinical Microbiology and Infections*.

[7] Harris R. L., Musher D. M., Bloom K. (1987). Manifestations of sepsis. *Archives of Internal Medicine*.

[8] Fourrier F., Chopin C., Goudemand J. (1992). Septic shock, multiple organ failure, and disseminated intravascular coagulation. *Chest*.

[9] Aygen B., Inan M., Doğanay M., Keleştimur F. (1997). Adrenal functions in patients with sepsis. *Experimental and Clinical Endocrinology & Diabetes: Official Journal, German Society of Endocrinology [and] German Diabetes Association*.

[10] Mayer J., Hajek R., Vorlicek J., Tomiska M. (1995). Sepsis and septic shock. *Supportive Care in Cancer*.

[11] Saeedi P., Halabian R., Fooladi A. A. I. (2019). Mesenchymal stem cells preconditioned by staphylococcal enterotoxin B enhance survival and bacterial clearance in murine sepsis model. *Cytotherapy*.

[12] Castro-Manrreza M. E., Montesinos J. J. (2015). Immunoregulation by mesenchymal stem cells: biological aspects and clinical applications. *Journal of Immunology Research*.

[13] Mei S. H. J., Haitsma J. J., Dos Santos C. C. (2010). Mesenchymal stem cells reduce inflammation while enhancing bacterial clearance and improving survival in sepsis. *American Journal of Respiratory and Critical Care Medicine*.

[14] Weil B. R., Markel T. A., Herrmann J. L., Abarbanell A. M., Kelly M. L., Meldrum D. R. (2009). Stem cells in sepsis. *Annals of Surgery*.

[15] McIntyre L. A., Stewart D. J., Mei S. H. J. (2018). Canadian critical care trials group the Canadian critical care translational biology group. Cellular immunotherapy for septic shock. A phase I clinical trial. *American Journal of Respiratory and Critical Care Medicine*.

[16] NCT03158727.

[17] NCT02883803.

[18] NCT03369275.

[19] Galstian G. M., Parovichnikova E. N., Makarova P. M. (2015). The results of the Russian clinical trial of mesenchymal stromal cells (MSCs) in severe neutropenic patients (pts) with septic shock (SS) (RUMCESS trial). *Blood*.

[20] NCT05283317.

[21] Schlosser K., Wang J.-P., Dos Santos C. (2019). Effects of mesenchymal stem cell treatment on systemic cytokine levels in a phase 1 dose escalation safety trial of septic shock patients^*∗*^. *Critical Care Medicine*.

[22] He X., Ai S., Guo W. (2018). Umbilical cord-derived mesenchymal stem (stromal) cells for treatment of severe sepsis: aphase 1 clinical trial. *Translational Research*.

[23] Pedrazza L., Lunardelli A., Luft C. (2014). Mesenchymal stem cells decrease splenocytes apoptosis in a sepsis experimental model. *Inflammation Research*.

[24] Xu J., Woods C. R., Mora A. L. (2007). Prevention of endotoxin-induced systemic response by bone marrow-derived mesenchymal stem cells in mice. *American Journal of Physiology - Lung Cellular and Molecular Physiology*.

[25] Wannemuehler T. J., Manukyan M. C., Brewster B. D. (2012). Advances in mesenchymal stem cell research in sepsis. *Journal of Surgical Research*.

[26] Jawad I., Lukšić I., Rafnsson S. B. (2012). Assessing available information on the burden of sepsis: global estimates of incidence, prevalence and mortality. *Journal of global health*.

[27] Kebriaei P., Robinson S. (2011). Mesenchymal stem cell therapy in the treatment of acute and chronic graft versus host disease. *Frontiers in Oncology*.

[28] Moemen M. E. (2012). Prognostic categorization of intensive care septic patients. *World Journal of Critical Care Medicine*.

[29] Abraham E., Laterre P.-F., Garg R. (2005). Drotrecogin alfa (activated) for adults with severe sepsis and a low risk of death. *New England Journal of Medicine*.

[30] Ranieri V. M., Thompson B. T., Barie P. S. (2012). Drotrecogin alfa (activated) in adults with septic shock. *New England Journal of Medicine*.

[31] Santamaria P. (2003). Cytokines and chemokines in autoimmune disease: an overview. *Advances in Experimental Medicine and Biology*.

[32] Ferrari G., Cusella-De Angelis G., Coletta M. (1998). Muscle regeneration by bone marrow-derived myogenic progenitors. *Science*.

[33] Yang J., Jia Z. (2014). Cell-based therapy in lung regenerative medicine. *Regenerative Medicine Research*.

[34] Noiseux N., Marquis-Gravel G., Mansour S., Shahzad U., Stewart D. J., Yau T. M. (2014). The current state of stem cell therapeutics: Canadian approaches in the international context. *Canadian Journal of Cardiology*.

